# Effects of CDT on Hemodynamics and Quality of Life in a Subgroup of Patients with Lower Limb Deep Vein Thrombosis Carel: A Case-Control Study

**DOI:** 10.1155/2022/6607240

**Published:** 2022-08-02

**Authors:** Kanghua Zhang, Jinlin Yan

**Affiliations:** ^1^Surgical Disinfection Supply Center, Ningbo Medical Center Lihuili Hospital, Ningbo City Zhejiang Province 315000, China; ^2^Vascular Surgery, The Affiliated People's Hospital of Ningbo University, Ningbo City Zhejiang Province 315000, China

## Abstract

**Objective:**

To explore the effects of combined catheter-directed thrombolysis (CDT) on hemodynamics and quality of life in a subgroup of patients with lower limb deep vein thrombosis carel by using a case-control study.

**Methods:**

Eighty-four patients with deep venous thrombosis (DVT: acute DVT and chronic DVT) of lower extremities treated in our hospital from April 2017 to June 2021 were randomly assigned into the control group (*n* = 42) and the research group (*n* = 42). The control group only received routine nursing combined with CDT; the research group was treated with cluster nursing l combined with CDT. The clinical efficacy, the difference in limb circumference, hemorheology, hemodynamics, coagulation index and life quality before and after treatment, and the nursing satisfaction scores were calculated. The effects of cluster nursing l combined with CDT on hemodynamics and life quality in patients with DVT of lower extremities were analyzed.

**Results:**

The clinical curative effect of the research group was better than that of the control group (*P* < 0.05). After intervention, the difference in the thigh and leg perimeter in the research group was reduced, and the difference in the thigh and leg perimeter in the research group was significantly lower than that in the control group (*P* < 0.05). After intervention, the whole blood low shear viscosity, plasma viscosity, platelet aggregation rate, and fibrinogen in the research group were lower than those in the control group (*P* < 0.05). After intervention, segmental venous volume (SVC), maximum venous blood flow (MVO), and SVC/MVO in the research group were significantly higher than those before intervention, VRT was significantly prolonged, and MVO and venous pressure recovery time (VRT) were significantly higher than those in the control group. After intervention, D-dimer and fibrinogen decreased, prothrombin time and activated partial thromboplastin time increased in the research group, and the improvement of blood coagulation index in the research group was significantly better than that in the control group (*P* < 0.05). After intervention, the scores of quality of life in the research group decreased, and the scores of physiological function, psychological function, social function, and health self-cognition in the research group were lower than those in the control group (*P* < 0.05). The satisfaction of patients in the research group was significantly higher than that in the control group (*P* < 0.05).

**Conclusion:**

The application of cluster nursing l combined with CDT can effectively prevent lower limb venous thrombosis after operation and can enhance patients' hemorheology, hemodynamics, and blood coagulation function and significantly promote their life quality, nursing satisfaction is high, and it is worth popularizing and applying in clinic.

## 1. Introduction

Lower extremity DVT (LEDVT) is a common vascular disease in the peripheral venous system, and its annual incidence is as high as 0.07%~0.14% [1]. It is the third cause of morbidity and death in cardiovascular diseases, seriously threatens human health, and increases medical expenses and the financial burden on patients.

Risk factors include advanced age, long-term bedridden immobilization, surgical trauma stress, tumor, pregnancy, and hormone therapy [1, 2]. The three most important factors that initiate thrombosis in human veins are blood stagnation, venous endothelial injury, and blood clotting [3]. The clinical manifestations are lower limb swelling, pain, decreased sensation and mobility, and aggravated symptoms after exercise. If there is no formal anticoagulant therapy in the acute stage, thrombus can spread gradually, from peripheral thrombus to complex thrombus (iliofemoral thrombus complex with peripheral thrombus), aggravating the pain and suffering of patients and even massive thrombus exfoliation and symptomatic pulmonary embolism leading to death [4]. A large sample epidemiological study of venous thromboembolism (VTE) reported that about 2.1%~4.7% of patients with pulmonary embolism (PE) in acute LEDVT died due to untimely treatment [2]. In the long term, the disease can develop into postthrombotic syndrome (PTS). The pathogenesis of PTS is not completely clear. It may come from venous hypertension caused by obstructive thrombosis and damage in venous intima and venous valve caused by acute thrombotic inflammation and eventually lead to chronic venous insufficiency [3]. The main clinical manifestations are lower limb swelling, pigmentation, lifestyle-restricted venous claudication, varicose veins, and venous ulcers. A lot of patients with DVT will have long-term complications, namely, PTS [4].

It has been reported that the life quality score of patients with PTS is comparable to that of patients with severe chronic diseases such as diabetes and congestive heart failure [5]. Anticoagulant therapy has always been the standard scheme recommended by some guidelines for the treatment of acute LEDVT [6]. However, even with the best anticoagulant therapy, there is also a high risk of PE and thrombosis recurrence, and the incidence of PTS after AC is as high as 48% [7]. Therefore, it is recommended in the latest guidelines that catheter-directed thrombolysis (CDT) can be used selectively for acute iliofemoral LEDVT, provided that the course of thrombosis is less than 2 weeks, there are no contraindications for thrombolysis, and the life expectancy is more than 1 year [8]. CDT can open the deep veins of the lower limbs at an early stage to prevent the recurrence of thrombosis and protect the structural integrity and normal function of the venous valves, thus reducing the incidence of PTS, especially in patients with iliofemoral deep vein thrombosis [9]. However, CDT still has many shortcomings, such as frequent monitoring of blood coagulation, ICU monitoring and treatment, long hospital stay, unbearable long prone position, potential intracranial hemorrhage, and the risks of massive hemorrhage of important organs. Therefore, more effective and safe auxiliary means of thrombus removal are needed.

Cluster nursing is a novel nursing model that provides targeted care to patients by educated and dedicated nurses who follow and cross-check a plan based on the patient's specific condition [9]. Cluster nursing is a group of nursing programs composed of three or more evidence-based measures that have been widely accepted in clinical practice. In the process of program implementation, each intervention must be continuously implemented, and one or more of them cannot be interrupted or selectively applied [10]. The purpose is to provide patients with the best medical and nursing services. In recent years, with the development of evidence-based nursing, cluster nursing is increasingly adopted to solve all kinds of nursing problems in clinical practice, which greatly promotes the development of cluster nursing. Cluster care is now widely used in clinical care, such as the management of chronic diseases, the prevention of ventilator-associated pneumonia, and the care of patients with malignancies and in intravenous line placement [10]. Xiaoxia et al. have reported that cluster nursing was carried out for elderly patients with lower limb fracture, which effectively reduced the incidence of complications such as pressure sore, pulmonary infection, VTE, and urinary system infection [11]. Some researchers carried out cluster nursing in the intensive care unit, which effectively reduced the incidence of iliofemoral venous catheter infection and indwelling iliofemoral venous catheter-related blood flow infection. Clinical practice has demonstrated that cluster nursing makes nurses' clinical decisions based on evidence; promotes the science, pertinence, and effectiveness of nursing measures; and enhances the outcome for patients [12, 13]. However, there are still many misunderstandings in the practice of clinical application of cluster nursing in our country. The biggest problem is that the name cluster nursing is applied, but its essence is not correctly understood. Cluster care is not a collection or simple patchwork of care measures but rather a translation of clinical guidelines or consensus into concrete clinical practice, incorporating the patient's wishes in order to improve patient outcomes. Based on this, 84 patients with DVT of lower extremities treated in our hospital from April 2017 to June 2021 were studied in this paper.

## 2. Patients and Methods

### 2.1. General Information

Eighty-four patients with LEDVT treated in our hospital from April 2017 to June 2021 were randomly assigned to the control group (*n* = 42) and the research group (*n* = 42). The control group only received routine nursing combined with CDT therapy. The research group was treated with cluster nursing l combined with CDT. In the research group, there were 25 males and 17 females, aged from 28 to 72 years, with an average age of 45.83 ± 13.66 years. The course of the disease was 5-30 days, with an average course of 17.62 ± 8.35 days. There were 23 cases of acute DVT (duration ≤ 14 d) and 19 cases of chronic DVT (duration > 30 d). There were 26 cases of left lower limb, 16 cases of right lower limb, 18 cases of iliofemoral type DVT, 20 cases of peripheral type DVT, and 14 cases of complex type DVT. There were 27 males and 15 females in the control group. Age ranged from 27 to 71 years with an average age of 44.63 ± 13.87 years, and there was no significant difference in age between the two groups. The course of disease was 3-30 d, with an average course of 16.37 ± 8.92 d. There were acute DVT20 in 22 cases, chronic DVT in 22 cases, left lower limb in 28 cases, right lower limb in 14 cases, iliofemoral type DVT in 16 cases, peripheral type DVT in 14 cases, and complex type DVT in 12 cases. There exhibited no significant difference in sex, age, course of disease, DVT site, and clinical classification (*P* > 0.05). This study was permitted by the Medical Ethics Association of our hospital, and all patients signed informed consent.

Selection criteria are the following: (1) in accordance with the diagnostic criteria made by the fourth academic meeting of the Chinese Society of Integrated Traditional Chinese and Western Medicine in 1995 [14], (2) age > 18 years, (3) no contraindications for thrombolysis, and (4) no severe compound injury and vascular and nerve injury.

Exclusion criteria are the following: (1) patients with a history of craniocerebral injury, cerebral infarction, or myocardial infarction in the past 3 months and patients with a history of bleeding in the digestive system and urinary system and a history of major surgery in the past 3 weeks; (2) patients with traumatic symptoms such as active bleeding or fractures; (3) patients with a history of severe hypertension, heart, liver, and kidney dysfunction and diabetes; (4) patients during pregnancy and puerperium; and (5) patients who fail to be treated in accordance with the regulations and affect the judgment of the curative effect.

### 2.2. Treatment Methods

#### 2.2.1. Admission-Related Examination and Basic Treatment

After admission, the patient was diagnosed according to medical history, signs, and US or CTV. The patient was examined to show the site of thrombus, the extent of involvement, vascular variation or malformation, blood routine, liver and kidney function, electrolyte, blood lipid, blood glucose, blood coagulation function, D-dimer, preinfusion examination, routine defecation, ECG, chest X-ray, abdominal vein and large vessel color ultrasound, cardiac ultrasound, and so on. Patients received absolute bed rest and limb elevation to avoid fatal PE and reduce limb swelling. Patients received anticoagulant sodium of low molecular weight heparin (6000 u/branch, subcutaneous injection, Q12h) in order to control thrombus dilatation and received intravenous infusion of flavonoid tablets or sodium aescin to improve venous function.

#### 2.2.2. Treatment Method

Both groups received catheter contact thrombolytic therapy, and the patients were in the prone position. After 1% lidocaine local anesthesia took effect, 6F sheath was placed under ultrasound guidance (affected side popliteal vein, posterior tibial vein, or great saphenous vein). The Misgurnus anguillicaudatus guide wire and angiographic catheter were adopted to enter the inferior vena cava through the stenosis or occlusion segment of deep vein thrombosis, and the catheter was removed and predilated into the catheter with a balloon (7 mm or 8 mm). Then, the 6F thrombolytic catheter was inserted into the thrombotic vein supported by the guide wire, the metal core at the end of the catheter was closed, and the catheter in the working area with lateral holes covered the whole thrombus. The catheter was connected to a micropump and was infused with urokinase (1.2 × 10^4^ U·kg^−1^·d^−1^) and maintained with heparin for 24 hours. Venous DSA examination of the affected limb was performed daily to evaluate the grade of thrombolysis. For daily monitoring of blood routine and blood coagulation function, when fibrinogen is less than 1.5 g/l, reduce the dosage of urokinase; when activated partial prothrombin time was more than 3 times or fibrinogen was less than 1 g/l, stop thrombolytic therapy and continue anticoagulation therapy (low molecular weight heparin calcium injection 6000 IU/Q12h). If postoperative reexamination of DSA revealed iliofemoral vein stenosis or iliac vein compression syndrome, immediately dilate the narrow segment of vein balloon (diameter 7 mm or 8 mm MUSTANGGH Boston Scientific, USA) expansion; if the stenosis is still greater than 50% after repeated dilatation, a large number of collateral circulation is open, or many contrast media are retained, stent implantation is performed in the diseased segment (12-14 mm in diameter Wallstent, Boston Scientific, USA).

#### 2.2.3. Nursing Intervention Measures

The control group received routine nursing, and the nursing staff routinely did rounds on time, taking the body temperature of patients on time. On the basis of the control group, the research group received cluster nursing: (1) the education and training of nurses are strengthened to understand the prevention process, nursing measures, and effects of venous thrombosis in detail and strictly implement the assessment system, etc., to enhance the sense of responsibility of nurses; (2) the nursing staff assessed the risk of the patients after admission, told them to stay in bed for those who were at risk of lower limb venous thrombosis, actively communicated with the patients to understand their inner thoughts, patiently tell the cause and harm of lower limb venous thrombosis and do a good job in positive prevention, timely dredge its negative psychology, and give psychological comfort and support; (3) the nursing staff made a healthy diet plan for the patients, told them to ban smoking and alcohol, and closely observed the changes of their vital signs and the bleeding of the access site, so as to help the patients turn over regularly. The pain and swelling of the lower extremities were evaluated and actively dealt with, and intermittent inflation-related devices could be used to prevent the patients with high risk; (4) the nursing staff should strengthen the analgesic nursing of the patients after the operation, replenish the water and electrolyte in time, avoid lower limb infusion and pressurized infusion, especially repeated venipuncture, dilute the drugs that stimulate the blood vessels of the body, and carry out drug prevention to observe whether there is bleeding; and (5) the nurses were educated about the CDT procedures, following a specific control program for each patient, did careful information and education, and looked for bleeding sites (nose, gingiva, vagina, access site, etc.).

### 2.3. Observation Index

#### 2.3.1. Evaluation Standard of Curative Effect

After nursing, the clinical efficacy was evaluated in accordance with the evaluation criteria established in Reference [15]. Cure: standing 20~30 min, there was no obvious swelling pain and heaviness and tenderness after 1500 m walking; lower limb edema subsided obviously or completely; compared with the healthy side, the circumference difference was less than 2 cm, and the blood vessels were completely recanalized by color Doppler vascular imaging. Significant effect: standing or walking 15~20 min, pain and swelling were significantly enhanced after 1000 m walking; lower limb edema was significantly relieved; compared with the healthy side, the circumference difference was less than 3 cm; in color Doppler vascular imaging, most of the blood vessels were recanalized. Effective: standing for 10 min, pain and swelling were promoted after 500 m walking; lower limb edema was alleviated, and the circumference difference was slightly reduced compared with the healthy side; a small part of blood vessels were recanalized by color Doppler vascular imaging. Ineffective: after treatment, the symptoms were not strengthened, or the edema of the affected limb was aggravated or complicated with PE. Total effective rate = (cure + effective + effective)/total number of cases × 100%.

#### 2.3.2. Clinical Symptoms

The change of swelling degree was evaluated by the circumference difference of bilateral thigh and calf. The 15 cm on the superior edge of the patella is the circumference of the thigh, and the 10 cm under the trochanter of the tibia is the circumference of the leg. Circumference difference = the circumference of the affected limb − the circumference of the healthy limb.

#### 2.3.3. Hemorheological Index

Whole blood low shear viscosity, plasma viscosity, platelet aggregation rate, and fibrinogen were detected by an automatic hemorheological detector before and after treatment.

#### 2.3.4. Hemodynamic Index

Segmental venous volume (SVC), maximum venous blood flow (MVO), and venous pressure recovery time (VRT) of all patients before and after treatment were measured by ultrasound, and the patency of deep vein was evaluated by the MVO/SVC value. MVO/SVC > 0.6 was regarded as deep venous patency, 0.5-0.6 as suspected thrombosis, and <0.5 as DVT.

#### 2.3.5. Blood Coagulation Function

Before and after intervention, fasting venous blood 2 ml was collected and placed in the anticoagulation tube, and the serum was separated by centrifugation. The levels of prothrombin time (PT), activated partial thromboplastin time (APPT), fibrinogen (Fib), and plasma D-dimer (D-dimer) were detected by latex immune turbidimetry.

#### 2.3.6. Quality of Life Scale

The self-designed life quality scale consists of four subscales, which are physical, psychological, social, and health self-awareness, with a total of 29 items. Cronbach's *α* coefficient of the scale is 0.79-0.91. The scale was scored by 1-5 grades. The lower the score, the higher the satisfaction.

#### 2.3.7. Satisfaction Survey

A hospital self-made satisfaction questionnaire was employed to evaluate patients' nursing satisfaction, which included five dimensions: physical care, receiving information, support, respect, and nursing flow. The full score is 100; the higher the score, the higher the satisfaction.

### 2.4. Statistical Analysis

The data were analyzed by SSPS21.0 statistical software, and the rate of qualitative data such as cause of injury and sex was presented (%). The quantitative data such as coagulation function and hemodynamics were compared by the *χ*^2^ test, and the quantitative data such as coagulation function and hemodynamics were presented by the mean ± standard deviation (*x* ± *s*). *P* < 0.05 indicated that the differences exhibited statistically significant.

## 3. Results

### 3.1. Comparison of Clinical Efficacy between the Two Groups

First of all, we compared the clinical effects. The research group was cured in 18 cases, markedly effective in 14 cases, effective in 9 cases, and ineffective in 2 cases, and the effective rate was 95.24%, while that in the control group was cured in 5 cases, markedly effective in 18 cases, effective in 14 cases, and ineffective in 5 cases, and the effective rate was 88.10%. The clinical curative effect of the research group was better compared to the control group (*P* < 0.05). All the results are indicated in Figure 1.

### 3.2. Comparison of Circumference Difference of Big Leg and Lower Leg between the Two Groups before and after Intervention

There was no significant difference in the circumference of the thigh and calf before and after the intervention (*P* > 0.05). After intervention, the circumference difference of the thigh and calf decreased. Compared with the control group, the circumference difference of the thigh and calf of the research group was significantly lower (*P* < 0.05). All the results are indicated in Table 1.

### 3.3. Comparison of Hemorheological Indexes between the Two Groups before and after Intervention

We compared the hemorheological indexes before and after intervention. Before intervention, there exhibited no significant difference in hemorheological indexes (*P* > 0.05). After intervention, all the indexes were lower than those before treatment. The whole blood low shear viscosity, plasma viscosity, platelet aggregation rate, and fibrinogen in the research group were lower compared to the control group (*P* < 0.05). All the results are indicated in Table 2.

### 3.4. Comparison of Hemodynamic Indexes between the Two Groups before and after Intervention

We compared the hemodynamic indexes before and after intervention. Before intervention, there exhibited no significant difference in hemodynamic indexes (*P* > 0.05). After intervention, SVC, MVO, and SVC/MVO were significantly higher compared to those before intervention, and VRT was significantly prolonged. Compared with the control group, MVO and VRT in the research group were significantly higher or longer (*P* < 0.05); the values of SVC and MVO/SVC in the control group were also higher, with no significant difference between the two groups (*P* > 0.05). All the results are indicated in Table 3.

### 3.5. Comparison of Blood Coagulation Function between the Two Groups before and after Intervention

We compared the blood coagulation function before and after intervention, and there exhibited no significant difference before intervention (*P* > 0.05). After intervention, D-dimer and Fib decreased, while PT and APTT increased. The improvement of blood coagulation indexes in the research group was significantly better compared to the control group (*P* < 0.05). All the results are indicated in Table 4.

### 3.6. Comparison of Life Quality Scores

We compared the scores of life quality. Before treatment, there exhibited no significant difference (*P* > 0.05). After treatment, the scores of life quality decreased. Compared between the two groups, the scores of physiological function, psychological function, social function, and health self-cognition in the research group were lower compared to the control group (*P* < 0.05). The results of all the data are indicated in Table 5.

### 3.7. Satisfaction Comparison

We compared the satisfaction scores, and the satisfaction scores of patients in the research group in physical care, receiving information, support, respect, and nursing process were significantly higher compared to the control group (*P* < 0.05). All the data results are indicated in Figure 2.

## 4. Discussion

Deep venous thrombosis (DVT) is defined as venous reflux disorder caused by abnormal coagulation of blood in deep veins [15]. It often occurs in the lower extremities and is the third largest vascular disease after cerebrovascular and coronary artery diseases. The incidence rate in Europe and the United States is about 0.1%. In recent years, the incidence of DVT is increasing year by year in China [16]. At present, DVT and PE are classified as venous embolism (VTE). It is considered that DVT and PE are clinical manifestations of venous embolism in different stages of the disease [17]. The main clinical manifestations of LEDVT are swelling, pain, dyskinesia, and increased muscle tone of the affected limb. Without timely intervention treatment, thrombus shedding along with the ascending blood circulation can lead to PE. Some PE is even fatal, and the site of lower limb DVT is more likely to have PE at the proximal end than at the distal end [18]. Therefore, a small number of patients with LEDVT were admitted to hospital with PE symptoms such as chest tightness, shortness of breath, chest pain, dyspnea, and hemoptysis. In addition, patients with DVT of lower extremities will also have postthromboembolic syndrome (PTS), which can cause long-term pain and blood stasis, affect normal life and working ability, and even lead to disability. It is also the main complication of DVT of lower extremities [19].

Clinically, according to the onset time of lower limb DVT, it is assigned into the acute phase, subacute phase, and chronic phase; the acute phase refers to the onset time within 14 days; the subacute phase refers to the onset time of more than 14 days, but not more than 30 days; the chronic phase refers to the onset time of more than 30 days [20]. The key step in the treatment of lower limb DVT is to open blocked blood vessels as soon as possible to restore blood flow. Failure to seek medical attention may result in the acute phase developing into a subacute or chronic phase, with the clot gradually organizing and not being easily dissolved by thrombolytic drugs [21]. Organized thrombus can cause changes in pulmonary blood flow if it adheres to the walls of pulmonary arteries and eventually develop into chronic thrombotic pulmonary hypertension; if it adheres to the walls of deep veins of the lower extremities, it can destroy the venous valves of the lower extremities and lead to venous valvular insufficiency of the lower extremities [21]. The treatment of acute lower limb DVT includes anticoagulation, thrombolytic therapy, surgical thrombectomy, and mechanical thrombectomy. Thrombolytic therapy is the main measure. In order to prevent the development of thrombus and distal branch venous thrombosis, anticoagulation is the basic treatment of lower limb DVT [22]. Thrombolytic therapy includes CDT and systemic venous thrombolysis. CDT is put into the DVT of the affected limb, and thrombolytic drugs can act on the thrombus directly, while systemic venous thrombolysis applies thrombolytic drugs to the whole body through the peripheral vein. The trauma of CDT is small, which reduces the influence on the function of the deep venous valve of lower extremities as much as possible, increases the opening of collateral branches, accelerates venous reflux, reduces intravenous pressure, and relieves edema and pain of lower extremities [23, 24]. Although CDT has many advantages, related complications may occur. Thus, it can be noticed that perioperative prevention is particularly important.

Although the clinic has paid more attention to the prevention of DVT, some preventive measures have been taken, but all of them are one-sided and do not form a systematic prevention strategy, and many preventive measures are only based on clinical experience without evidence-based scientific basis and the preventive effect on DVT [25]. Therefore, based on evidence, the establishment of a set of systematic, scientific, and targeted prevention strategies is of great significance to the prevention of DVT. At present, there are some studies on the prevention of DVT, including thrombus risk assessment and preventive measures. The 10th edition of the guidelines for antithrombotic treatment of VTE of the American College of Thoracic Physicians has pointed out that not all patients are suitable for prophylactic treatment of DVT [26]. Risk stratification should be carried out according to the risk assessment scale, and appropriate measures should be taken. Meanwhile, in view of the hidden and atypical characteristics of the occurrence of DVT, it is of great significance to evaluate the risk of DVT for the prevention of DVT [25, 26]. There are many methods to evaluate the risk factors for thrombus, including Caprini thrombus risk factor assessment, Padua score, Davison score, Autar score, RAPT score, and Well's score scale. Scholars have indicated that Well's DVT score combined with plasma D2 polymer detection can enhance the accuracy of DVT detection and is suitable for clinicians to diagnose DVT. RAPT is suitable for thrombus risk assessment of trauma patients, which is recommended by the expert consensus on screening and treatment of DVT in orthopedic trauma patients [26]. Thus, it can be noticed that different thrombus risk assessment tools have their own advantages and limitations. Patients should be assessed in the whole process, and follow-up and dynamic assessment should be made at any time according to the changes of the disease. According to the risk of patients, corresponding preventive measures should be taken to reduce the incidence of DVT.

The preventive measures of DVT include basic prevention, physical prevention, and drug prevention [27]. First, for basic prevention, it mainly includes paying attention to the protection of venous vessels of the affected limb in the process of operation, puncture, static therapy, and venous catheter maintenance, doing a good job of posture management, raising the affected limb, guiding patients to carry out perioperative functional exercise, getting out of bed as early as possible when the condition permits, providing health education on DVT-related knowledge to patients, and doing a good job in the control of basic diseases [27]. The effect of the above basic preventive measures has been confirmed by a number of clinical studies for a long time, which is worth affirming. However, there are the following problems in the clinical implementation of basic preventive measures: nurses do not receive unified training on DVT-related knowledge, do not have enough knowledge about DVT, cannot provide high-quality health education for patients, and cannot guarantee the homogenization of health education without unified training [26, 27]. The specific content, frequency, and intensity of functional exercise lack corresponding standards, and there are no unified requirements, which cannot guarantee the completion quality of patients' functional exercise; clinical nurses have a lot of work, and health education and functional exercise guidance are often unable to be carried out; health education lacks corresponding theoretical guidance, such as health belief model, knowledge, belief, and practice model, which leads to the scientific nature and effect of health education being not good [28]. Therefore, how to implement the basic preventive measures of DVT in order to achieve the best preventive effect is worthy of further discussion.

Clinical practice demonstrates that cluster nursing provides nurses with evidence for clinical decision-making; enhances the science, pertinence, and effectiveness of nursing measures; and improves the outcome of patients. The results of this study indicated that the clinical curative effect of the research group was better compared to the control group (*P* < 0.05). The circumference difference of large leg and calf in the research group exhibited significantly lower compared to the control group (*P* < 0.05). The whole blood low shear viscosity, plasma viscosity, platelet aggregation rate, and fibrinogen in the research group were lower compared to the control group (*P* < 0.05). After intervention, MVO and VRT in the research group were significantly higher or longer compared to the control group (*P* < 0.05); the values of SVC and MVO/SVC in the control group were also higher compared to the control group, but with no statistical significance (*P* > 0.05). The improvement of blood coagulation indexes in the research group was significantly better compared to the control group (*P* < 0.05). The scores of physiological function, psychological function, social function, and health self-cognition in the research group were lower compared to the control group (*P* < 0.05). The satisfaction scores of patients in the research group were significantly higher compared to the control group in terms of physical care, receiving information, support, respect, and nursing process (*P* < 0.05). It demonstrates that the application of cluster nursing is beneficial to promote the hemodynamics and blood coagulation function of the patients and significantly enhance their quality of life. The education and training of nursing staff and the implementation of strict assessment and reward and punishment system can not only strengthen their sense of responsibility but also strengthen their professional and practical skills in the prevention of venous thrombosis of lower extremities. And it can actively assess the risk of patients after hospitalization, urge patients to stay in bed, and inform them of the knowledge about lower limb venous thrombosis. All play a significant role in the prevention of lower extremity venous thrombosis. Nursing staff can help patients to turn over and give analgesia nursing and timely supplement of electrolytes, which can reduce lower limb swelling, pain, and vasospasm caused by pain and strengthen drug prevention. It is helpful to reduce the probability of lower limb venous thrombosis and enhance the quality of life such as physiological function. Nursing staff should give psychological comfort, timely dredge their negative psychology, reduce their worries, improve their bad psychological state, formulate a reasonable diet plan for patients, and strictly ban smoking and alcohol, which all play a role in enhancing the condition of patients and promote their quality of life. We analyzed the reasons for better clinical outcomes in cluster nursing as follows.

First is physical prevention, including periodic inflatable pressurization system (IPC), plantar vein pump (VFP), grade elastic socks (GCS), and other methods. After eliminating contraindications, IPC, VFP, and GCS can promote venous and lymphatic reflux of lower extremities, increase blood flow velocity, reduce venous stasis, and achieve the purpose of preventing DVT without increasing the incidence of PE. Some studies have indicated that IPC, VFP, and GCS can effectively reduce the incidence of DVT, and the effect of combined use is better [27, 28]. However, Lu et al. pointed out that the preventive effect of the combination of the above physical prevention methods was not better compared to its alone [28]. Therefore, the effect of single or combined use of clinical physical prophylaxis remains to be further demonstrated by clinical research, and there is no final conclusion.

Second is drug prevention, mainly the use of a variety of anticoagulants, including subcutaneous injection of low molecular weight heparin or oral anticoagulants such as rifampicin, warfarin, and aspirin. The 2016 edition of “Guidelines for the Prevention of VTE in Chinese Orthopaedic Surgery” recommended that the most commonly used anticoagulants in the perioperative period of orthopedic surgery are low molecular weight heparin and Xa factor inhibitor rivaroxaban [29]. Some studies have confirmed that the use of anticoagulants such as low molecular weight heparin and rivaroxaban can effectively reduce the incidence of DVT [29, 30]. Low molecular weight heparin is adopted by subcutaneous injection, which has the advantages of safety and low risk of bleeding, but platelet count needs to be monitored when there is a bleeding tendency. Rivaroxaban is a new oral anticoagulant with the advantages of easy to use and good compliance of patients. But severe renal insufficiency is taboo. Some studies have indicated that there is no statistical difference in the efficacy and safety of the two drugs in the prevention of DVT. Weiwen and other scholars [30] also found that low molecular weight heparin and rivaroxaban have little effect on the prevention of postoperative DVT, and there is no statistical significance (*P* = 0.09). To sum up, the use of basic prevention, physical prevention, and drug prophylaxis alone can reduce the incidence of DVT. However, in recent years, comprehensive prevention has gradually become the consensus of some experts and has been recommended by a number of authoritative evidence-based guidelines.

At present, cluster nursing is widely adopted in many fields of clinical nursing, such as the prevention and control of nosocomial infection, the management of chronic diseases, the prevention of ventilator-associated pneumonia, the nursing of acute and critically ill patients, the nursing of patients with malignant tumors, and the application in intravenous catheterization [30]. Shiyuan et al. carried out cluster nursing measures of accelerated rehabilitation surgery for patients with thyroid cancer, which effectively relieved the pain of the patients, shortened the indwelling time of the drainage tube, reduced the number of cases of postoperative postural syndrome, reduced the incidence of postoperative complications, shortened the length of stay in hospital, and greatly promoted the rehabilitation of the patients [31]. Some researchers carried out cluster nursing in the intensive care unit, which effectively reduced the incidence of iliofemoral venous catheter infection and indwelling iliofemoral venous catheter-related bloodstream infection. Some studies indicate that cluster nursing for patients with acute pancreatitis with enteral nutrition can effectively reduce the incidence of enteral nutrition-related complications, enhance the nutritional status of patients, and shorten the duration of hospitalization [32]. There are some limitations in this study. First, the sample size of this study is not large, and it is a single-center study, so bias is inevitable. In future research, we will carry out multicenter, large-sample prospective studies, or more valuable conclusions can be drawn.

Conclusively, the combined application of cluster nursing on the basis of CDT therapy can significantly reduce the risk of lower limb venous thrombosis, lower limb swelling, and lower limb pain in hand patients after operation and has a better preventive effect on lower limb venous thrombosis. It can significantly enhance the quality of life of patients, promote their hemodynamic indexes, and strengthen their nursing satisfaction, which is worthy of clinical promotion.

## Figures and Tables

**Figure 1:** Comparison of clinical efficacy between the two groups.

**Figure 2:** Comparison of nursing satisfaction between the two groups.

**Table 1:** Comparison of circumference difference of large leg and lower leg between the two groups ($\bar{x}\pm s$).

Grouping	*N*	Thigh circumference difference		Calf circumference difference	
		Before intervention	After intervention	Before intervention	After intervention
Control group	42	5.88 ± 3.44	2.79 ± 0.83^a^	4.24 ± 2.36	2.78 ± 1.22^a^
Research group	42	6.27 ± 3.21	2.23 ± 0.37^b^	4.51 ± 2.17	2.14 ± 0.95^b^
*t* value		0.537	3.994	0.546	2.682
*P* value		>0.05	<0.05	>0.05	<0.05

Note: comparison before and after intervention in the control group, ^a^*P* < 0.05; comparison of research group before and after intervention, ^b^*P* < 0.05.

**Table 2:** Comparison of hemorheological indexes in two groups ($\bar{x}\pm s$).

Grouping	*N*	Whole blood low shear viscosity (mPa·s)		Plasma viscosity (mPa·s)		Platelet aggregation rate (%)		Fibrinogen (g/l)	
		Before intervention	After intervention	Before intervention	After intervention	Before intervention	After intervention	Before intervention	After intervention
Control group	42	12.13 ± 2.51	10.83 ± 1.81^a^	2.26 ± 0.36	1.71 ± 0.33^a^	65.95 ± 9.03	60.88 ± 8.42^a^	5.46 ± 1.34	4.14 ± 0.97^a^
Research group	42	12.34 ± 2.33	9.51 ± 1.66^b^	2.17 ± 0.38	1.91 ± 0.35^b^	66.81 ± 8.72	56.08 ± 7.43^b^	5.65 ± 1.42	3.34 ± 0.92^b^
*t* value		0.397	3.483	1.114	2.269	0.444	2.770	0.631	3.878
*P* value		>0.05	<0.05	>0.05	<0.05	>0.05	<0.05	>0.05	<0.05

Note: comparison before and after intervention in the control group, ^a^*P* < 0.05; comparison of research group before and after intervention, ^b^*P* < 0.05.

**Table 3:** Comparison of hemodynamic indexes between the two groups ($\bar{x}\pm s$).

Grouping	*N*	SVC (ml)		MVO (ml)		MVO/SVC		VRT (s)	
		Before intervention	After intervention	Before intervention	After intervention	Before intervention	After intervention	Before intervention	After intervention
Control group	42	5.82 ± 1.94	7.36 ± 2.74^a^	2.91 ± 1.73	6.08 ± 2.55^a^	0.46 ± 0.23	0.79 ± 0.25^a^	12.26 ± 4.05	8.66 ± 3.54^a^
Research group	42	5.76 ± 1.83	8.19 ± 2.83^b^	2.81 ± 1.63	7.74 ± 2.35^b^	0.45 ± 0.21	0.88 ± 0.23^b^	13.78 ± 4.43	7.22 ± 1.18^b^
*t* value		0.146	1.366	0.272	3.102	0.208	1.717	1.641	2.501
*P* value		>0.05	>0.05	>0.05	<0.05	>0.05	<0.05	>0.05	<0.05

Note: comparison before and after intervention in the control group, ^a^*P* < 0.05; comparison of research group before and after intervention, ^b^*P* < 0.05.

**Table 4:** Comparison of blood coagulation function between the two groups ($\bar{x}\pm s$).

Grouping	*N*	D-dimer (mg/l)		PT (s)		APTT (s)		Fib (g/l)	
		Before intervention	After intervention	Before intervention	After intervention	Before intervention	After intervention	Before intervention	After intervention
Control group	42	4.67 ± 1.08	3.66 ± 0.52^a^	9.21 ± 1.04	10.54 ± 1.11^a^	23.62 ± 2.01	29.08 ± 2.12^a^	5.23 ± 0.87	4.68 ± 0.52^a^
Research group	42	4.72 ± 1.05	2.23 ± 0.41^b^	9.24 ± 1.03	12.08 ± 1.22^b^	23.64 ± 2.03	35.64 ± 2.15^b^	5.21 ± 0.88	3.71 ± 0.44^b^
*t* value		0.215	13.995	0.133	6.051	0.045	14.080	0.105	9.229
*P* value		>0.05	<0.05	>0.05	<0.05	>0.05	<0.05	>0.05	<0.05

Note: comparison before and after intervention in the control group, ^a^*P* < 0.05; comparison of research group before and after intervention, ^b^*P* < 0.05.

**Table 5:** Comparison of life quality scores between the two groups ($\bar{x}\pm s$, points).

Grouping	*N*	Physiological function		Psychological function		Social function		Healthy self-cognition	
		Before intervention	After intervention	Before intervention	After intervention	Before intervention	After intervention	Before intervention	After intervention
Control group	42	15.47 ± 4.68	13.98 ± 2.13^a^	16.55 ± 3.57	14.43 ± 4.47^a^	18.74 ± 3.15	16.92 ± 2.61^a^	15.54 ± 3.19	13.86 ± 1.95^a^
Research group	42	15.93 ± 4.41	11.54 ± 2.61^b^	16.43 ± 3.88	10.94 ± 1.46^b^	18.56 ± 3.69	12.57 ± 3.29^b^	15.65 ± 3.38	10.49 ± 2.71^b^
*t* value		0.464	4.694	0.147	4.810	0.240	6.713	0.153	6.542
*P* value		>0.05	<0.05	>0.05	<0.05	>0.05	<0.05	>0.05	<0.05

Note: comparison before and after intervention in the control group, ^a^*P* < 0.05; comparison of research group before and after intervention, ^b^*P* < 0.05.

## Data Availability

No data were used to support this study.
